# Synergistic Effect of Conventional Medicinal Herbs against Different Pharmacological Activity

**DOI:** 10.1155/2022/7337261

**Published:** 2022-06-29

**Authors:** Huma Ali, Daoud Ali, Bader O. Almutairi, Gokhlesh Kumar, Gizachew Assefa Karga, Chandran Masi, Venkatesa Prabhu Sundramurthy

**Affiliations:** ^1^Department of Chemistry Maulana Azad National Institute of Technology, Bhopal, India; ^2^Department of Zoology, College of Science, King Saud University, P.O. Box 2455, Riyadh 11451, Saudi Arabia; ^3^Clinical Division of Fish Medicine, University of Veterinary Medicine Vienna, 1210 Vienna, Austria; ^4^Addis Ababa Science and Technology University, Addis Ababa, Ethiopia; ^5^Bioprocess and Biotechnology, Center of Excellence, Addis Ababa Science and Technology University, P.O. Box 16417, Addis Ababa, Ethiopia; ^6^Department of Chemical Engineering, College of Biological and Chemical Engineering, Addis Ababa Science and Technology University, P.O. Box 16417, Addis Ababa, Ethiopia

## Abstract

*Triticum aestivum* (Family: Poaceae), *Ocimum sanctum* (Family: Lamiaceae), and *Tinospora cordifolia* (Family: Menispermaceae) are commonly known as wheatgrass, tulsi, and giloy, respectively, which are the plants used as medicines for the treatment of various diseases. All three medicinal plants possess phenolic compounds with other important chemical constituents such as polysaccharides, aliphatic compounds, and alkaloids. The extract of these plants has been prepared and investigated for antioxidant, total phenolic content, total flavonoid content, and antimicrobial study in order to discover potential sources for new pharmaceutical formulations. To determine the antioxidant activity, a free radical scavenging assay for 2,2-diphenyl-1-picrylhydrazyl (DPPH) and hydrogen peroxide was performed using ascorbic acid as the standard. The *R*^2^ value of the prepared extract was found to be 0.9964 and 0.990 in DPPH and hydrogen peroxide scavenging activity, respectively. The phenolic and flavonoid content was found to be 87.50 *μ*l/ml and 58.00 *μ*l/ml, respectively. The diffusion method was used to screen the antimicrobial activity of the prepared extract sample against various microorganisms. This extract showed better results for antioxidant and antimicrobial activity.

## 1. Introduction

Multidrug therapy is a useful method that focuses on inhibiting or destroying harmful agents (such as cancer cells or infections) as well as activating human body defense or healing mechanisms. It is the result of the progressive abandonment of the previously held dogma of monodrug therapy; for decades, pharmacological research was predicated on the discovery of a single active principle [1]. In terms of phytotherapy research, traditional Chinese medicine, Ayurveda, and traditional Western phytomedicines have just recently begun to be scientifically validated and valued. Furthermore, over the last 20 years, the use of conventional drugs in combination with complementary and alternative medicine (CAM) has increased worldwide, including not just homoeopathy, naturopathy, chiropractic, and energy medicine but also ethnopharmacology and phytotherapy [2]. Many diseases now have a complicated aetiology that could be treated more effectively with a drug combination strategy rather than a single administration. In Western countries, efficient multidrug therapy is routinely used to treat multifactorial or complicated disorders (e.g., cancer, hypertension, metabolic and inflammatory diseases, acquired immune deficiency syndrome (AIDS), and infections) [3].

Synergistic effects are the combined effects of at least two drugs that have a greater influence than either of them could have had individually. It is what happens when chemical substances or biological structures interact, resulting in a larger overall effect than the sum of their separate effects. Skin damage caused by combining tobacco smoke and UV radiation is more noticeable than tobacco smoke alone or UV radiation alone, as an example of synergistic effects. The liver is harmed by both carbon tetrachloride and ethanol (ethyl liquor) [4]. When used combined, they cause more serious liver damage than the sum of their individual effects on the liver. Barbiturate medications can have more harmful effects on the central nervous system (CNS) when combined with general anaesthetics, alcohol (acute consumption), narcotic analgesic (pain reliever), and other sedative-hypnotic agents (by causing CNS depression), when doctors use ampicillin and gentamicin to treat bacterial heart infections. This is done because the two antimicrobials target different parts of the bacteria, and combining them destroys the microscopic organisms faster, allowing for speedier recovery. Another example of synergism is the treatment of cancer. Chemotherapy and radiation therapy are often administered to cancer patients. They work to halt cancer cell proliferation by focusing on distinct aspects of the replicating process [5].

Social insects are an example of synergy in ecology since they have diverse responsibilities and classes in their colony. Chemical signals picked up by their antennae are the primary means by which they communicate with one another. *Colobopsis explodens*, for example, exhibits an intriguing trait known as autothysis. While wrapped around their victim, these ants will spontaneously erupt (thus the name). This suicidal gesture is a desperate attempt to protect their nest. Soldier termites will rupture their bodies to function as a roadblock to tunnels, preventing invaders from entering their nest, which is known as autothysis [6, 7].

*Myxococcus xanthus*, a predatory myxobacterial species, exhibits cooperative behaviour that leads to synergism. *M. xanthus* is a bacterium that feeds on other bacteria in the soil. Through the soil, they create a cooperative hunting group (colony). As they come into contact with bacteria and feed on it, they emit digestive enzymes. They can feed a much larger prey and generate considerably more digestive enzymes in colonies than they do individually, which has the disadvantage of being distributed through the soil [8, 9] (Figure 1).

Pest synergy is defined as the presence of two or more parasites in the same host. As an example, the presence of two different types of parasitic worms would result in synergistic negative effects that are significantly bigger than the impacts of each individual parasitic worm. As a result, the impact is proportional to the density. Even in infection, this is visible. The host that harbours pathogenic bacteria or viruses may or may not produce symptoms of infection, as the impact of the pathogens' presence is determined by the size or population density of the pathogens [10].

Since ancient times, we have used plants as major sources of medicines and antidotes. Compounds derived from plants (i.e., phytochemicals) are an enormous interest of researchers as natural alternatives to synthetic or chemical-based compounds [11]. The Indian System of Medicine is based on the use of plant extracts to treat various diseases. The Indian subcontinent features a diverse flora and fauna in a relatively small geographic region due to topography, altitude, and climate changes [12]. It therefore also contains an impressive amount of medical plants. Over 3000 plant species have medicinal properties in India. Most of the wild varieties found here are rich in medicinal properties like antibacterial, antiviral, antihelminthic, anticancer, sedative, laxative, cardiotonic, and diuretic. According to the World Health Organization (WHO), any plant that possesses therapeutic (curative) properties or exerts a beneficial pharmacological (relating to drugs) effect on the animal body is called a medicinal plant [13].

It has now been discovered that the pharmacological activity (i.e., drug-like activity) of a plant is because they can naturally synthesize secondary metabolites (small organic molecules which are unnecessary for their growth, development, or reproduction), like oils, glycosides, vitamins, alkaloids, and tannins. Metabolite plants produce a vast range of organic substances that can be divided into two categories: primary and secondary metabolites. Primary metabolites, unlike secondary metabolites, play a direct role in normal growth, development, and reproduction. Ethanol, lactic acid, and some amino acids are all examples of primary metabolites. Secondary metabolites have complex structures and extraordinary concentrations in their cells [14]. They are unique to a specific species. They are identified by highly specific actions within or outside the cells. They are often produced as by-products of primary metabolism, perhaps to deal with excess metabolic compounds and play an important role in plant defense. Thousands of plants worldwide are used to cure various diseases, like cancer and many chronic diseases, including cardiovascular diseases (diseases related to the heart and circulatory system). Traditional medicinal plants contain antiviral properties and are used to treat viral infections in both animals and humans [15].

## 2. Materials and Methods

### 2.1. Plant Material and Preparation of Combined Sample of Extract

25 g grass of *Triticum aestivum* (Poaceae), 15 g stem of *Tinospora cordifolia* (Menispermaceae), and 10 g of leaves of *Ocimum sanctum* (Labiatae) were collected from a botanical garden of Bhopal, Madhya Pradesh, India, and authenticated. Plant materials were washed, dried, powdered, and then extracted by using solvent methanol and acetone in the ratio of 70 : 30, ethyl acetate and acetone, respectively, for 24 hours. 50 ml of each extract was mixed to form a combined sample of extract (Figure 2).

### 2.2. Chemicals

Sigma Chemical Co. provided the 2,2-diphenyl-1-picrylhydrazyl (DPPH), Folin-Ciocalteu reagent, ascorbic acid and gallic acid, and sodium nitrite (L-AA) (St. Louis, MO, USA). Other chemical reagents were available commercially and were of analytical quality.

### 2.3. Screening of Antioxidant Activity of Combined Sample of Extract

#### 2.3.1. 2,2-Diphenyl-2-picryl-hydrazyl (DPPH) Radical Scavenging Assay

The delocalization of the extra electron above the molecule as a whole distinguishes the DPPH molecule as an established free radical. The molecules then do not dimerise, as they would with mainly more free radicals. The deep violet colour owes to delocalization in ethanol solution, which is characterised by an absorption band at about 517 nm [16].

Different concentrations of combined sample of extract were arranged for DPPH radical scavenging activity. The dilutions (400 to 1000 l/ml) were then varied with 0.5 ml DPPH solution and incubated for 30 minutes in the dark at room temperature. Using the formula below, the % inhibition test was calculated. Using distilled water as a blank, absorbance was measured at 517 nm [17, 18].

(1) $$\begin{array}{c} \%\text{inhibition of DPPH radical}=\frac{\text{Control}-\left(\text{sample with DPPH}-\text{sample without DPPH}\right)}{\text{Control}}\times 100. \end{array}$$

#### 2.3.2. Hydrogen Peroxide Radical Scavenging (H_2_O_2_) Assay

Certain variations were used to test the ability of combined sample of extract to scavenge hydrogen peroxide. At varying concentrations of aq. arranged extract (400 to 1000 l/ml), 0.5 ml of hydrogen peroxide solution made in phosphate buffer saline with a pH of 7.4 was added. After 10 minutes, the absorbance was measured at 230 nm against a blank solution containing phosphate buffer but no hydrogen peroxide. For background subtraction, a single blank sample was used for each concentration. The absorbance of hydrogen peroxide without the extract sample was measured at 230 nm as a control. The following formula was used to compute the % inhibitory activity. As a standard, gallic acid (10-100 g/ml) was used [19].

(2) $$\begin{array}{c} \%\text{inhibition of }{\text{H}}_{2}{\text{O}}_{2}\text{ radical}=\frac{\text{Control}-\left(\text{sample with }{\text{H}}_{2}{\text{O}}_{2}-\text{sample without }{\text{H}}_{2}{\text{O}}_{2}\right)}{\text{Control}}\times 100. \end{array}$$

#### 2.3.3. Total Flavonoid Content (TFC)

Flavonoids can scavenge virtually all known ROS depending on their structure [20]. TFC was performed using a 1 l/ml extract concentration and rutin as a reference. The absorbance of a mixture was measured at 510 nm versus produced water as a blank using the method of Zou et al. [21].

#### 2.3.4. Total Phenolic Content (TPC)

The total phenolic content of the combined sample of extract was determined using the Folin-Ciocalteu reagent, as described by McDonald et al. As a control, gallic acid was utilised [22].

### 2.4. Screening of Antimicrobial Activity of Combined Sample of Extract

#### 2.4.1. Test Microorganisms

The bacterial strains *Escherichia coli* (MTCC No. 1698), *Proteus* (MTCC No. 658), *Staphylococcus aureus* (MTCC No. 9886), *Staphylococcus cohnii* (MTCC No. 10219), and *Klebsiella pneumoniae* (MTCC No. 3040) were selected based on their scientific and medicinal importance. All the strains were purchased from the Institute of Microbial Technology, Chandigarh, and used for evaluating antimicrobial activity.

#### 2.4.2. Growth Media Preparation

Nutrient agar for bacterial strains was prepared according to the following standard procedure.

#### 2.4.3. Nutrient Agar

*(1) Purpose*. Nutrient agar is a nutrient agar that can be used to grow a wide range of nonfastidious bacteria. It was created in response to a demand for a standardized media for the study of water and wastewater, dairy products, and diverse meals.

*(2) Method for Preparation*. In 250 ml filtered water, dissolve 6 g of the powder. Boil for 1 minute with frequent agitation to completely dissolve the powder. Autoclave for 15 minutes at 121°C. Cool to 45-50 degrees Celsius. Fill sterile 20 ml glass universal tubes with 15-20 ml of the supplied media. Allow thirty minutes for the tubes to freeze before resting them leaning at 30-60°C to achieve the slope effects. The sterility of the media was confirmed by incubating it at 37°C for 24 hours and then storing it at 40°C for up to two weeks.

Composition of nutrient agar media used was as follows:

- Peptone: 5 g/l
- Beef extract: 1.50 g/l
- Yeast extract: 1.50 g/l
- Sodium chloride: 5.0 g/l
- Distilled water: 1000 ml

#### 2.4.4. Determination of Antimicrobial Activity

The nutrient agar media was sterilised by autoclaving for 15 minutes at 121°C and 15 pounds of pressure. Petri dishes were filled with sterile media. A 5 mm diameter cork bearer was used to bore the cemented plates. The antimicrobial experiments were conducted on plates having wells. Antibacterial activity of 0.1 ml of the above produced combined sample of extract at varied concentrations of 7%, 5%, 3%, and 1% was tested against Gram-positive *S. aureus* and *S. cohnii* and Gram-negative *E. coli*, *Proteus*, and *K. pneumoniae*. The well diffusion method [23] was used to demonstrate this.

The streak plate method was used to inoculate the prepared culture plates with several bacteria strains. With a 6 mm cork borer, wells were drilled into the medium surface. Using a sterile syringe, the various samples were poured into the well. For bacterial activity, the plates were incubated at 37°C for 24 hours. Each concentration of the several samples was put to the test against a different microbe. The zone of inhibition was estimated by adding the well diameter to the diameter of the inhibition zone around the well (in mm). The average values of the readings were calculated in four separate fixed directions.

## 3. Results

### 3.1. Antioxidant Activity

Line of regression was found to be *y* = 0.0564*x* + 26.984 (3) and *y* = 0.0854*x* + 12.773 (4) which revealed IC_50_ to be 435.91 and 408.08 *μ*l/ml in the above prepared extract sample for 1,1-diphenyl-2-picryl-hydrazyl (DPPH) radical and hydrogen peroxide (H_2_O_2_) scavenging assay, respectively. It was observed that inhibition of DPPH and H_2_O_2_ was increasing continuously. Thus, from 400 *μ*l/ml to 1000 *μ*l/ml, the *R*^2^ value was found to be 0.9964 and 0.9904, respectively, which could be considered as the best fit one. Degradation of H_2_O_2_ showed the decline in absorbance of H_2_O_2_ radical at 230 nm caused by reaction between antioxidants present in the prepared extract and free radical (Figures 3–5 and Tables 1–3).

The total phenols were expressed as *μ*l/ml gallic acid equivalent using the standard curve equation: *y* = 0.016*x* + 0.119, *R*^2^ = 0.981 (5).  Figure 6 shows the variation of mean absorbance with concentration of gallic acid.  Table 4 shows the contents of total phenols that were measured by Folin-Ciocalteu reagent in terms of gallic acid equivalent. The phenolic content was found to be 87.500 *μ*l/ml.

The total flavonoids were expressed as *μ*g/mg rutin equivalent using the standard curve equation: *y* = 0.002*x* + 0.011, *R*^2^ = 0.994 (6).  Figure 7 shows the variation of mean absorbance with concentration of rutin.  Table 5 shows the contents of flavonoid in terms of rutin equivalent that was found to be 58.00 *μ*l/ml.

### 3.2. Antimicrobial Activity

The zone of inhibition obtained in the present study was mentioned in mean ± SD. The antibacterial activity of the prepared extract sample of different concentration was analyzed against different bacterial strains. The better activity was observed in this combined sample of extract against different microorganism (Table 6).

## 4. Discussion

1,1-Diphenyl-2-picrylhydrazyl (DPPH), is a type of established organic radical. The DPPH oxidative assay is used worldwide in the quantification of antioxidant activity. The ability of natural reagents to scavenge the DPPH radical can be stated as its extent of antioxidation capability [24]. The colour of an alcoholic solution of DPPH is deep purple, with an absorption peak at 517 nm that fades when the radical scavenger is present in the immediate system and when the odd electron of the nitrogen in DPPH is paired [25]. The produced extract was tested for linear inhibition of DPPH in the concentration range of 400-1000 g/ml in this study.

Several oxidase enzymes and activated phagocytes produce hydrogen peroxide *in vivo*, and it is known to have a role in the death of diverse tissues. There is growing evidence that hydrogen peroxide can operate as a messenger molecule in the creation and activation of numerous inflammatory mediators, either directly or indirectly via its reduction product, OH- [26]. When a scavenger is treated with H_2_O_2_, the loss of H_2_O_2_ can be evaluated using a peroxidase test method. The prepared combined sample of extract was evaluated in this study to see if it had considerable hydrogen peroxide scavenging capability.

Phenolic compounds are a group of antioxidant agents which acts as free radical terminators. Estimation of the total phenolic content revealed that the prepared extract possesses good total phenolic and flavonoid content. Total phenol content was estimated on the basis of gallic acid. Results are mentioned as gallic acid equivalent (GAE). Total flavonoid was expressed in rutin equivalent (RE). Prepared extract showed positive results against all microorganisms. These finding are due the synergistic effect of individual extract of *Triticum aestivum*, *Ocimum sanctum*, and *Tinospora cordifolia.*

## 5. Conclusion

According to the findings of this study, the above-mentioned combined sample of extract has the potential to be used as medication because it contains antioxidant and antimicrobial properties. To fully validate the established claim, additional knowledge of contemporary pharmaceutical techniques such as extraction and separation of active chemical constituents is required. In order to determine its position in medical claims, additional, well-controlled double-blind trial exams are required to reconsider the efficacy and side effects.

## Figures and Tables

**Figure 1:** *Myxococcus xanthus*: synergy by cooperation.

**Figure 2:** Flowchart showing preparation of combined sample of extract.

**Figure 3:** Effect of ascorbic acid for antioxidant activity using DPPH as free radical scavenging agent.

**Figure 4:** Effect of prepared extract sample for antioxidant activity using DPPH as free radical scavenging agent.

**Figure 5:** Effect of prepared extract sample for antioxidant activity using H_2_O_2_ as free radical scavenging agent.

**Figure 6:** Standard curve of gallic acid.

**Figure 7:** Standard curve of rutin.

**Table 1:** Effect of ascorbic acid for antioxidant activity using DPPH as free radical scavenging agent.

% inhibition	Intercept (*C*)	Slope (*M*)	IC_50_ (*μ*l/ml)
50	41.655	0.033	253.03

**Table 2:** Effect of prepared extract sample for antioxidant activity using DPPH as free radical scavenging agent.

% inhibition	Intercept (*C*)	Slope (*M*)	IC_50_ (*μ*g/ml)
50	26.984	0.0564	435.91

**Table 3:** Effect of prepared extract sample for antioxidant activity using H_2_O_2_ as free radical scavenging agent.

% inhibition	Intercept (*C*)	Slope (*M*)	IC_50_ (*μ*g/ml)
50	12.773	0.0854	408.08

**Table 4:** Total phenolic content of prepared extract sample.

Extract sample (*μ*l/ml)	Absorbance	Gallic acid equivalent (*μ*l/ml)
1000	1.51	87.50

**Table 5:** Total flavonoid content of the prepared extract.

Extract (*μ*l/ml)	Absorbance	Rutin equivalent (*μ*l/ml)
1000	0.156	58.00

**Table 6:** Zone of inhibition at different concentrations of prepared extract sample against different microorganism.

Prepared extract sample					
Conc.	Zone of inhibition mm in diameter (mean ± SD)				
	*Escherichia coli*	*Proteus*	*Staphylococcus aureus*	*Staphylococcus cohnii*	*Klebsiella pneumoniae*
7%	16.54 ± 0.32	21.54 ± 0.35	20.78 ± 0.49	19.38 ± 0.21	22.45 ± 0.26
5%	16.09 ± 0.21	19.87 ± 0.28	19.45 ± 0.43	18.76 ± 0.32	21.65 ± 0.87
3%	15.67 ± 0.60	18.98 ± 0.19	18.23 ± 0.62	17.91 ± 0.76	19.98 ± 0.54
1%	14.12 ± 0.98	18.03 ± 0.16	17.11 ± 1.45	17.01 ± 2.43	18.54 ± 0.89

## Data Availability

The original contributions presented in the study are included in the article; further inquiries can be directed to the corresponding author.
